# Protein-Specific Prediction of RNA-Binding Sites Based on Information Entropy

**DOI:** 10.1155/2022/8626628

**Published:** 2022-10-03

**Authors:** Yue Ji, Lu Bai, Menglong Li

**Affiliations:** ^1^College of Chemistry, Sichuan University, Chengdu, Sichuan 610064, China; ^2^Product R&D and Testing Center, Shilin Xingdian Agricultural Products Development Co., Ltd., Kunming, Yunnan 652200, China

## Abstract

Understanding the protein-RNA interaction mechanism can help us to further explore various biological processes. The experimental techniques still have some limitations, such as the high cost of economy and time. Predicting protein-RNA-binding sites by using computational methods is an excellent research tool. Here, we developed a universal method for predicting protein-specific RNA-binding sites, so one general model for a given protein was constructed on a fixed dataset by fusing the data of different experimental techniques. At the same time, information theory was employed to characterize the sequence conservation of RNA-binding segments. Conversation difference profiles between binding and nonbinding segments were constructed by information entropy (IE), which indicates a significant difference. Finally, the 19 proteins-specific models based on random forest (RF) were built based on IE encoding. The performance on the independent datasets demonstrates that our method can obtain competitive results when compared with the current best prediction model.

## 1. Introduction

RNA-binding proteins (RBPs) play an important role in gene expression and regulation since they are highly involved in various biological processes such as mRNA stability [1], stress responses [2], and gene regulation at the transcriptional and posttranscriptional levels [3]. Understanding RNA-protein interactions can lead to further study on the mechanisms underlying these biological processes. Accurate identification of RNA-protein binding sites is very useful for studying these biological processes. In recent years, many high-throughput experimental methods are useful for studying these biological processes. In recent years, many high-throughput experimental methods, such as PAR-CLIP [4], have been developed which can accurately determine the binding sites of RNA-protein interactions at the experimental level. However, these experimental methods are time-consuming and cost-effective. It is necessary to develop computational methods to predict the binding sites between RNAs and proteins.

At present, several researchers have developed computational methods for predicting RNA-protein binding sites. RNA context is a method with sequence and accessibility information to predict binding motifs [5], and Maticzka et al. present GraphProt to predict binding preferences by using RNA sequence and secondary structural contexts [6]. Zhang et al. integrate RNA sequence, secondary structural contexts, and RNA tertiary structural information by using a deep learning framework for modeling structural binding preferences and predicting binding sites of RBPs [7]. Strazar et al. develop an integrative orthogonality-regularized nonnegative matrix factorization (iONMF) to predict RBP interaction sites on RNAs [8]. In iONMF, the features of protein-RNA interactions are the positions of RNA structure and sequence motifs, RBP cobinding, and gene region types. Pan et al. have given iDeep, iDeepS, and iDeepE to predict RNA-protein binding sites from RNA sequences [9]. iDeep developed a novel hybrid convolutional neural network and deep belief network with RNA sequence, secondary structure, clip-cobinding, region type, and motif features to predict the RBP interaction sites and motifs on RNAs. iDeepS can identify the binding sequence and structure motifs from RNA sequences at the same time by using convolutional neural networks and a bidirectional long short-term memory network only with RNA sequence and predicted secondary structure. iDeepE improves the network structure to predict RNA-protein binding sites and motifs by combining local and global deep convolutional neural networks.

The above research has achieved satisfactory prediction results, and some of them obtain the high area under curve (AUC) values in most datasets, such as iDeepS. However, there are still limitations deserving improvement in previous studies, including different experimental datasets and the selection of features.

Since different experimental methods for the same protein are usually different, previous prediction methods are all based on different datasets from different experimental techniques, so multiple different models are usually constructed for a given protein, such as the protein ELAVL1 which has two datasets with different protocols of PAR-CLIP and CLIP-seq [10, 11]. We know that each protein has a definite RNA-binding motif, but there may be some errors that make the RBPs undetectable during the experiment. Different protocols can make up for the loss caused by experimental errors, so different experimental datasets for a given protein could be merged as one general dataset to build a protein-specific model which is universal to different experimental techniques. In addition, the current accuracy of the predicted secondary structures is relatively low, so the reported performance may be of some discount for the existing methods based on the predicted secondary structures.

In our study, we developed a simpler and universal model for predicting RNA-protein binding sites for different proteins only based on RNA sequence information. Firstly, for 19 proteins, 19 general protein-specific datasets were achieved by fusing different experimental data. Then, only based on the sequence information, k-mer-based features and IE profiles were respectively used to represent the binding segments. Finally, the RF model based on IE profiles was proved to be with the best performance, compared with 3, 4, and 5-mer features. The final model yields satisfactory results with an average AUC of 0.849 for the 19 proteins. In addition, the model that uses single RNA secondary structures was also built, but it gives the lowest prediction accuracy. Overall, our method only based on sequence conservation information by IE can obtain competitive results when compared with the current best prediction model.

## 2. Materials and Methods

### 2.1. Dataset

We downloaded the datasets from iDeepS [12] which is available at https://github.com/xypan1232/iDeepS. iDeepS collected the data from iONMF [8], and it contains 31 CLIP-seq datasets with 19 binding proteins. Original CLIP-seq data are from servers iCount (http://icount.biolab.si) and DoRiNA [13]. In the iDeepS datasets, protein-RNA-binding sites are positive samples. Fifty bases were selected from each side of the binding site by sliding window to form a sequence with a length of 101. Genes that had never been identified as interacting sites in 31 experiments were used as negative samples.

In our work, in order to construct the protein-specific and experiment-universal model, we merged 31 CLIP-seq datasets into 19 general datasets for 19 different proteins. Here, due to the different structures, Ago2-MNase and Ago2, as well as ELAVL1-MNase and ELAVL1, are deemed as different proteins from each other [14]. Finally, we separated each dataset into training and testing one according to the ratio of 5 : 1. The detailed information about the 19 datasets is shown in Table 1.

### 2.2. Methods

#### 2.2.1. Feature Extraction

Here, we tried to represent protein binding RNAs from RNA primary sequences by IE profiles and K-mer features. Besides, since RNA secondary structures have been used and demonstrated to be useful for representing binding segments by previous reports [15], they were also extracted to be compared with features from sequence information.

*(1) Information Entropy*. Information entropy (IE) was proposed by Shannon [16] and has been deemed as one of the simplest and most common measures of conservation at a site on protein sequences in the field of bioinformatics [17]. IE describes the occurrence probability of discrete random events, and it also reflects the evolutionary conservatism of each location in the sequence. It has been successfully used in our previous research works of Shi et al. [18] and Wang et al. [19]. Shi et al. used IE to distinguish the difference between methylated and nonmethylated peptide segments, and Wang et al. used it to classify Type IV secreted effectors from the negative sample based on the N-terminal 100 residues.

In our work, IE is used to measure evolutionary conservation differences between binding and nonbinding sites of RNA sequences. The information content of each nucleic base at each position can be calculated as the input features to predict protein-RNA interaction binding sites.

*(2) K-mer*. K-mer is a common genomic feature in bioinformatics, and it has been widely used to identify some regions in biological DNA or protein molecules. Zhang et al. use K-mer to predict piRNA [20], and Cao et al. make use of K-mer to predict subcellular localization of lncRNA [21]. To characterize protein binding RNA sequences, we used all the 3–5 nt strings, including 3mer strings, 4mer strings, and 5mer strings.

*(3) RNA Secondary Structure*. RNA secondary structure refers to the planar structure formed by various components, such as single-stranded region structure, stem-ring structure, and double-stranded structure, which are composed of complementary base pairs in an RNA molecule and self-folding through these structures. RNA secondary structure is a kind of reversal formed by RNA molecules under natural conditions.

RNA secondary structures are widely used in protein-RNA-binding site prediction, such as iONMF [8] and iDeepS [22]. RNAshapes is a tool for predicting the secondary structure of RNA [23]. We used RNAshapes to obtain RNA secondary structure annotations by referring to Fukunaga et al. [24]. In this way, we can obtain the secondary structure of each position in the sequence (Figure 1). Six types of secondary structures were considered, including stems (S), multiloops (M), hairpins (H), internal loops (I), dangling end (T), and dangling start (F).

#### 2.2.2. Random Forests

The random forests (RFs) algorithm is an integrated classification model [25]. Its construction process is mainly composed of three aspects: the generation of a training set, the construction of a decision tree, and the generation of the algorithm. First, we need to generate training sets from the original data by sampling. Through the bagging algorithm, N samples are extracted from the original data set. Each sample will produce a decision tree, and the generated decision tree does not need pruning, thus establishing N decision trees to form forests.

At present, the RF algorithm is one of the most popular machine learning algorithms, and it has been widely used to solve biological classification [26–30].

The RF model we used in this study was implemented by a random forest package in the *R* language.

#### 2.2.3. Evaluation Indicators

We used five effective performance evaluation indicators to evaluate the predictive ability of the model, namely area under curve (AUC), sensitivity (SE), specificity (SP), accuracy (ACC), and Matthew's correlation coefficient (MCC), respectively. AUC represents the area under the receiver operating characteristic (ROC) curve. When drawing the ROC curve, the true positive is taken as ordinate, and the false positive is taken as abscissa. The closer the AUC is to 1, the better the prediction will be these metrics are commonly defined as follows:

(1) $$\begin{array}{c} SE=\frac{TP}{TP+FN}\text{,}\\ \begin{array}{c} SP=\frac{TN}{TN+FP},\\ \begin{array}{c} ACC=\frac{TP+TN}{TP+TN+FP+FN},\\ MCC=\frac{\left(TP+TN\right)-\left(FP+FN\right)}{\sqrt{\left(TP+FP\right)\left(TP+FN\right)\left(TN+FP\right)\left(TN+FN\right)}}, \end{array} \end{array} \end{array}$$

where TP, FP, TN, and FN are true positive, false positive, true negative, and false negative, respectively.

## 3. Results and Discussion

### 3.1. Difference Analysis between Positive and Negative Samples

The distribution of nucleic bases is the basic information for an RNA sequence. With the segment length of 101 bases, we plotted two sample logos [15, 31] of 19 protein training sets to show the difference in base composition between positive and negative samples in each dataset. Here, we select two of them as examples. We can find that the positive and negative samples of the same protein have obvious differences in base compositions. For each segment, the 51st base in the positive sample sequence is the protein-RNA interaction site. According to the literature [32], the binding motif of protein-RNA interaction is usually 6–8 bases. From Figure 2(a), we can find that the (Figure 2) base locations of 48–54 in positive samples are obviously enriched with A and T. Negative samples were not enriched with A and T. Similarly, for the MOV10 data set, we can find that the 48–54 base positions of positive samples have obvious C and G enrichment from Figure 2(c). Especially at the 51st position of the positive sample, there was a significant C base enrichment. Negative samples do not have the above observations. Thus, the difference in base composition between positive and negative samples is significant.

We also plotted the two sample logos of the secondary structure of 19 protein training sets and showed the difference in the secondary structure of positive and negative samples for each data set. When protein and RNA interact, they both have unique space structures [33]. Therefore, the secondary structure of positive and negative samples will be different. It is also proved by our two sample logos. In Figure 2(b), we can find that the 48–54 positions in the positive samples of QKI datasets are usually multiloop (M) and hairpin (H). In the secondary structure of negative samples, we find that there are more stem (S) structures. In Figure 2(d), the positive sample of the MOV10 dataset is stem (S) structures at 48–54 positions. Negative samples did not show many stem (S) structures. We can also find that the positive and negative samples have obvious secondary structure differences by using two sample logos.

Then, we calculated the information entropy of 19 datasets. Information entropy can characterize the evolutionary conservation of each position in a sequence. We selected two training datasets of PUM2 and TIA1 to show the results of IE difference between positive and negative samples in Figure 3. From Figure 3, we can find that the IE values of positive and negative samples have obvious differences. We know that the lower the IE value of a given position is, the more conservative this position is. In general, we can easily see that all bases in the positive dataset are more conservative than those in the negative dataset. Moreover, there are significant conservation differences between positive and negative samples at the location of the 51st base and its adjacent bases, as marked by the red ovals in Figure 3.

The large difference in sequence conservativeness between binding and nonbinding sequences means that IE will be an important feature for predicting potential protein-RNA interaction sites.

### 3.2. Results on the Original 31 Datasets and the Combined 19 Datasets

According to the definition of IE and IG, we calculated the IG value of each position in the sequence. The IG value can quantitatively reflect the evolutionary conservation of each site in the sequence. We can find that the evolutionary conservatism of positive and negative samples is obviously different. Firstly, we use a single IG as the feature to construct the classifying model.  Figure 4 shows the AUC of 31 original test sets. The average AUC value of test datasets is 0.86, which indicates that IE is generally effective for predicting binding sites of protein-RNA interactions.

In order to get a more general model, we merged the datasets from different experiments for the same protein, so 19 protein-specific datasets were achieved. According to 19 proteins, the protein-specific model for each protein was constructed on each protein-specific dataset.  Figure 5 shows the AUCs of the combined test datasets, and Table 2 lists the detailed information. We can find that IE-based models also yield good prediction performance with an average AUC of 0.807. Moreover, 12 of 19 models give the AUC values higher than 0.8. The results of test datasets indicate that the general prediction model for each protein is valid, and it is a feasible way to develop the protein-specific model for the data from different experiments.

Secondly, six protein training sets were selected from 19 proteins according to the results of the model constructed with a single information entropy feather.  Table 3 shows the AUC comparison of three models based on the features of *K* = 3, 4, and 5, respectively. The result of 4-mer is similar to that of 5-mer and better than that of 3-mer. When *K* = 5, the feature dimension is 1028, so there are many positions in 1028 features with a result of 0. In order to reduce the noise of the model, we give up 5-mer as a feature. Finally, we chose *K* = 4.

Previous research has selected secondary structures as a feature to predict protein-RNA interaction binding sites [7]. We also tried to introduce the secondary structure into our prediction model.  Table 4 is the test sets AUC of the original 31 datasets using the secondary structure separately. However, we find that the contribution of a single secondary structure to the model is very small. The average AUC is only 0.55. There are specific secondary structures when proteins interact with RNA. But the RNA secondary structure used in current research is not the real secondary structure. They are derived from predictive tools such as RNAshapes [23] and RNAfold [34]. So, it will provide some wrong information to the model. Because the secondary structure cannot provide a positive impact on the prediction performance of the model, we do not choose to add the secondary structure to the final prediction model.

### 3.3. Comparison of Our Work and Other's works

Finally, we construct a hybrid model to predict protein-RNA interaction binding sites by combining IE with 4-mer. Then, the two models constructed by us with IE and IE + 4-mer were compared with the reported tool of iDeepS [12].  Table 5 shows the comparisons among the three models. On average, the hybrid model based on IE + 4-mer is superior to the model only with IE. For most datasets, the prediction performance of the hybrid model is almost equal to that of iDeepS. The average AUC of our hybrid model is 0.849, and that of iDeepS is 0.863. However, iDeepS is a tool based on sequence and secondary structure information. Our hybrid model is only sequence information. So, it is more concise and practical.

The prediction performance of the models constructed with information entropy and 4-mer feather across 31 original experiment datasets can be seen in Table 6. The detailed comparison results are shown in Table 5.

## 4. Conclusions

In this work, we have developed a simpler and more applied model for predicting protein-RNA interaction binding sites. According to the same binding protein, we merged the original datasets from different experiments, so the model constructed by the merged dataset is more general. We compared the performance of the prediction models with single IE, K-mer, and RNA secondary structures, respectively, and we found that models based on single IE and single 4-mer give satisfactory performance. Then, we constructed a hybrid model based on IE + 4-mer and compared it with the reported tool of iDeepS. We find that our hybrid model gives a competitive performance. However, in this paper, we first develop a general model for a specific protein, and our model is only based on the sequence information, so it is more feasible than other tools based on RNA structures.

## Figures and Tables

**Figure 1:** Conversion diagram of RNA secondary structure.

**Figure 2:** A two-sample logo to show position-specific distribution difference of base and secondary structure between binding and nonbinding sequence. (a) The difference of base in the QKI dataset; (b) the difference of secondary structure in the QKI dataset; (c) the difference of base in the MOV10 dataset; and (d) the difference of secondary structure in the MOV10 dataset.

**Figure 3:** Comparison of conservation in each position between binding and nonbinding sequence through Information entropy value.

**Figure 4:** The AUCs of single information entropy feather across 31 original experiment datasets.

**Figure 5:** The AUCs of single information entropy feather across 19 merged experiment datasets.

**Table 1:** The prediction performance of the models constructed with a single information entropy feather across 31 original experiment datasets.

Training groups	Protein	SE	SP	ACC	MCC	AUC_train	AUC_test
A	1 Ago/EIF	0.500	0.504	0.502	0.004	0.605	0.583
	3 Ago2-1	0.523	0.444	0.490	−0.032		0.623
	4 Ago2-2	0.515	0.548	0.528	0.062		0.656
	5 Ago2	0.473	0.508	0.489	−0.019		0.554
B	6 eIF4AIII-1	0.745	0.845	0.795	0.593	0.851	0.858
	7 eIF4AIII-2	0.780	0.805	0.793	0.585		0.873
C	8 ELAVL1-1	0.860	0.118	0.501	−0.033	0.750	0.715
	10 ELAVL1A	0.763	0.119	0.460	−0.153		0.626
	11 ELAVL1-2	0.869	0.090	0.501	−0.065		0.703
D	12 ESWR1	0.870	0.735	0.803	0.611	0.858	0.896
E	13 FUS	0.885	0.855	0.870	0.740	0.916	0.914
	14 Mut FUS	0.890	0.840	0.865	0.731		0.912
F	15 IGFBP1-3	0.690	0.675	0.683	0.365	0.628	0.771
G	16 hnRNPC-1	0.595	0.840	0.718	0.449	0.947	0.830
	17 hnRNPC-2	0.685	0.835	0.760	0.526		0.844
H	18 hnRNPL-1	0.680	0.750	0.715	0.431	0.754	0.810
	19 hnRNPL-2	0.740	0.730	0.735	0.470		0.805
	20 hnRNPL-like	0.625	0.710	0.668	0.336		0.732
I	21 MOV10	0.960	0.535	0.748	0.547	0.776	0.835
J	22 Nsun2	0.685	0.745	0.715	0.431	0.832	0.796
K	23 PUM2	0.920	0.795	0.858	0.721	0.887	0.915
L	24 QKI	0.840	0.890	0.865	0.731	0.920	0.937
M	25 SRSF1	0.705	0.795	0.750	0.502	0.785	0.848
N	26 TAF15	0.885	0.855	0.870	0.740	0.906	0.930
O	27 TDP-43	0.815	0.845	0.830	0.660	0.819	0.889
P	28 TIA1	0.760	0.875	0.818	0.639	0.999	0.900
	29 TIAL1	0.645	0.840	0.743	0.494		0.842
Q	30 U2AF2	0.780	0.855	0.818	0.637	0.901	0.903
	31 U2AF2 (KD)	0.700	0.865	0.783	0.573		0.874
R	2 Ago2-MNase	0.239	0.659	0.451	−0.113	0.605	0.405
S	9 ELAVL1-MNase	0.719	0.245	0.491	−0.040	0.605	0.499

**Table 2:** The prediction performance of the models is constructed with a single information entropy feather across 19 merged experiment datasets.

Training groups	SE	SP	ACC	MCC	AUC_train	AUC_test
A	0.635	0.607	0.621	0.217	0.639	0.659
B	0.765	0.820	0.793	0.465	0.847	0.865
C	0.734	0.708	0.721	0.368	0.777	0.792
D	0.870	0.735	0.803	0.482	0.858	0.896
E	0.885	0.848	0.866	0.557	0.916	0.914
F	0.690	0.675	0.683	0.312	0.628	0.771
G	0.640	0.838	0.739	0.400	0.947	0.837
H	0.682	0.730	0.706	0.347	0.754	0.783
I	0.960	0.535	0.748	0.447	0.776	0.835
J	0.685	0.745	0.715	0.360	0.832	0.796
K	0.920	0.795	0.858	0.550	0.887	0.915
L	0.840	0.890	0.865	0.556	0.920	0.937
M	0.705	0.795	0.750	0.410	0.785	0.848
N	0.885	0.855	0.870	0.561	0.906	0.930
O	0.815	0.845	0.830	0.513	0.819	0.889
P	0.700	0.865	0.783	0.458	0.999	0.874
Q	0.743	0.860	0.801	0.479	0.901	0.888
R	0.239	0.659	0.451	−0.113	0.605	0.405
S	0.719	0.245	0.491	−0.040	0.605	0.499

**Table 3:** AUCs of 6 selected proteins with a single K-mer.

Protein	AUC of 3-mer	AUC of 4-mer	AUC of 5-mer
QKI	0.9	0.899	0.919
U2AF2	0.871	0.8871	0.886
SRSF1	0.853	0.856	0.867
Mut FUS	0.829	0.836	0.841
Nsun2	0.76	0.763	0.767
IGFBP1-3	0.657	0.675	0.686

**Table 4:** The prediction performance of the models is constructed with a single secondary structure feather across 31 original experiment datasets.

Training groups	Protein	SE	SP	ACC	MCC	AUC train	AUC test
A	1 Ago/EIF	0.505	0.500	0.503	0.005	0.537	0.513
	3 Ago2-1	0.420	0.555	0.488	−0.025		0.509
	4 Ago2-2	0.440	0.580	0.510	0.020		0.510
	5 Ago2	0.530	0.420	0.475	−0.050		0.464
B	6 eIF4AIII-1	0.035	0.965	0.500	0.000	0.560	0.547
	7 eIF4AIII-2	0.350	0.745	0.548	0.103		0.600
C	8 ELAVL1-1	0.895	0.090	0.493	−0.025	0.632	0.498
	10 ELAVL1A	0.635	0.410	0.523	0.046		0.533
	11 ELAVL1-2	0.620	0.620	0.620	0.240		0.662
D	12 ESWR1	0.460	0.640	0.550	0.102	0.582	0.555
E	13 FUS	0.565	0.550	0.558	0.115	0.630	0.578
	14 Mut FUS	0.565	0.710	0.638	0.278		0.642
F	15 IGFBP1-3	0.565	0.710	0.638	0.278	0.523	0.642
G	16 hnRNPC-1	0.500	0.745	0.623	0.253	0.679	0.661
	17 hnRNPC-2	0.335	0.915	0.625	0.307		0.670
H	18 hnRNPL-1	0.540	0.500	0.520	0.040	0.573	0.551
	19 hnRNPL-2	0.505	0.600	0.553	0.105		0.564
	20 hnRNPL-like	0.465	0.510	0.488	−0.025		0.470
I	21 MOV10	0.440	0.580	0.510	0.020	0.521	0.520
J	22 Nsun2	0.615	0.530	0.573	0.146	0.610	0.595
K	23 PUM2	0.600	0.590	0.595	0.190	0.565	0.625
L	24 QKI	0.600	0.590	0.595	0.190	0.724	0.625
M	25 SRSF1	0.085	0.910	0.498	−0.009	0.522	0.464
N	26 TAF15	0.580	0.625	0.603	0.205	0.609	0.618
O	27 TDP-43	0.580	0.625	0.603	0.205	0.553	0.618
P	28 TIA1	0.155	0.955	0.555	0.183	1.000	0.636
	29 TIAL1	0.120	0.950	0.535	0.126		0.567
Q	30 U2AF2	0.120	0.950	0.535	0.126	0.602	0.567
	31 U2AF2 (KD)	0.330	0.705	0.518	0.038		0.548
R	2 Ago2-MNase	0.545	0.470	0.508	0.015	0.499	0.516
S	9 ELAVL1-MNase	0.485	0.550	0.518	0.035	0.519	0.506

**Table 5:** The comparison results among the model of single information entropy, the model of single information entropy with 4-mer, and iDeepS.

Protein	Information entropy	Information entropy + 4-mer	iDeepS
1 Ago/EIF	0.583	0.708	0.773
3 Ago2-1	0.623	0.832	0.865
4 Ago2-2	0.656	0.839	0.868
5 Ago2	0.554	0.592	0.634
6 eIF4AIII-1	0.858	0.932	0.950
7 eIF4AIII-2	0.873	0.934	0.953
8 ELAVL1-1	0.715	0.921	0.932
10 ELAVL1A	0.626	0.875	0.893
11 ELAVL1-2	0.703	0.907	0.919
12 ESWR1	0.896	0.904	0.917
13 FUS	0.914	0.936	0.934
14 Mut FUS	0.912	0.920	0.958
15 IGFBP1-3	0.771	0.709	0.717
16 hnRNPC-1	0.830	0.929	0.960
17 hnRNPC-2	0.844	0.966	0.975
18 hnRNPL-1	0.810	0.827	0.756
19 hnRNPL-2	0.805	0.802	0.769
20 hnRNPL-like	0.732	0.746	0.711
21 MOV10	0.835	0.839	0.813
22 Nsun2	0.796	0.811	0.835
23 PUM2	0.915	0.963	0.962
24 QKI	0.937	0.945	0.966
25 SRSF1	0.848	0.873	0.887
26 TAF15	0.930	0.934	0.964
27 TDP-43	0.889	0.913	0.930
28 TIA1	0.900	0.911	0.930
29 TIAL1	0.842	0.856	0.893
30 U2AF2	0.903	0.921	0.953
31 U2AF2 (KD)	0.874	0.891	0.931
2 Ago2-MNase	0.405	0.615	0.591
9 ELAVL1-MNase	0.499	0.566	0.613

**Table 6:** The prediction performance of the models is constructed with information entropy and 4-mer feather across 31 original experiment datasets.

Training groups	Protein	SE	SP	ACC	MCC	AUC_train	AUC_test
A	1 Ago/EIF	0.530	0.730	0.630	0.265	0.750	0.708
	3 Ago2-1	0.815	0.680	0.748	0.500	0.750	0.832
	4 Ago2-2	0.805	0.700	0.753	0.508	0.750	0.839
	5 Ago2	0.365	0.720	0.543	0.091	0.750	0.592
B	6 eIF4AIII-1	0.810	0.875	0.843	0.686	0.924	0.932
	7 eIF4AIII-2	0.870	0.835	0.853	0.705	0.924	0.934
C	8 ELAVL1-1	0.925	0.755	0.840	0.690	0.897	0.921
	10 ELAVL1A	0.850	0.755	0.803	0.608	0.897	0.875
	11 ELAVL1-2	0.890	0.720	0.805	0.619	0.897	0.907
D	12 ESWR1	0.850	0.800	0.825	0.651	0.845	0.904
E	13 FUS	0.870	0.875	0.873	0.745	0.895	0.936
	14 Mut FUS	0.830	0.885	0.858	0.716	0.895	0.920
F	15 IGFBP1-3	0.690	0.560	0.625	0.252	0.695	0.709
G	16 hnRNPC-1	0.865	0.850	0.858	0.715	0.952	0.929
	17 hnRNPC-2	0.960	0.870	0.915	0.833	0.952	0.966
H	18 hnRNPL-1	0.775	0.725	0.750	0.501	0.765	0.827
	19 hnRNPL-2	0.780	0.715	0.748	0.496	0.765	0.802
	20 hnRNPL-like	0.645	0.735	0.690	0.382	0.765	0.746
I	21 MOV10	0.875	0.655	0.765	0.543	0.793	0.839
J	22 Nsun2	0.725	0.735	0.730	0.460	0.832	0.811
K	23 PUM2	0.920	0.870	0.895	0.791	0.927	0.963
L	24 QKI	0.895	0.855	0.875	0.751	0.941	0.945
M	25 SRSF1	0.785	0.790	0.788	0.575	0.858	0.873
N	26 TAF15	0.870	0.890	0.880	0.760	0.897	0.934
O	27 TDP-43	0.750	0.875	0.813	0.630	0.888	0.913
P	28 TIA1	0.775	0.900	0.838	0.680	0.998	0.911
	29 TIAL1	0.645	0.875	0.760	0.534	0.998	0.856
Q	30 U2AF2	0.865	0.810	0.838	0.676	0.895	0.921
	31 U2AF2 (KD)	0.855	0.760	0.808	0.618	0.895	0.891
R	2 Ago2-MNase	0.545	0.625	0.585	0.171	0.605	0.615
S	9 ELAVL1-MNase	0.280	0.755	0.518	0.040	0.593	0.566

## Data Availability

The dataset can be accessed upon request.
